RETRACTED

# Diagnostic Efficacy of CT Radiomic Features in Pulmonary Invasive Mucinous Adenocarcinoma

**DOI:** 10.1155/2022/5314225

**Published:** 2022-06-25

**Authors:** Aizhu Sheng, Pengfei Zhou, Yizhai Ye, Keda Sun, Zhenhua Yang

**Affiliations:** ^1^Department of Radiology, Hwa Mei Hospital, University of Chinese Academy of Sciences, Zhejiang 315000, China; ^2^Department of Radiology, Ninghai First Hospital, Ningbo, Zhejiang 315600, China; ^3^Department of Radiology, No. 2 Hospital of Yinzhou District, Ningbo, Zhejiang 315100, China; ^4^Department of Thoracic Surgery, Hwa Mei Hospital, University of Chinese Academy of Sciences, Zhejiang 315000, China

## Abstract

In order to solve the problem of the effect of CT images on the diagnosis of lungs, the authors proposed a method for the diagnosis of invasive mucinous adenocarcinoma of the lungs based on CT radiomic features, and the modified method is found by reviewing past cases: among the 34 cases of primary pulmonary lymphoma, 12 cases were nodular mass type, 19 cases were nonnodular mass type, and 3 cases were mixed type; 13 cases involved bilateral lung lobes, 7 cases involved right lung, and 4 cases involved left lung example. There were 17 cases of tumor consolidation density shadow, 17 cases of mixed density shadow, the average CT value was about 32HU, 15 cases of cavitation sign, 6 cases of cavity, 9 cases of angiography sign, 30 cases of air bronchus sign, 22 cases of bronchiectasis, bronchial stenosis or amputation in 8 cases, pleural effusion in 12 cases, lymph node enlargement in 15 cases, and pleural metastasis in 2 cases. The final pathological results included 24 cases of membrane-associated lymphoid tissue (MALT) lymphoma, 9 cases of diffuse large B-cell lymphoma (DLBCL), and 1 case of T-cell lymphoma. The CT manifestations of primary pulmonary lymphoma (PPL) are diverse and do not have obvious specificity, the imaging manifestations are correlated with pathological types, and air bronchial signs, bronchiectasis, angiography signs, and other signs are used for the diagnosis of PPL. This is of great significance for the diagnosis of PPL.

## 1. Introduction

Lung cancer has become the malignant tumor with the highest morbidity and mortality in the world. In China, the incidence and mortality of lung cancer are increasing year by year, it has always been at the forefront, statistics from China's national cancer center show that there are about 800,000 new lung cancer patients in China every year, and 630,000 people died of lung cancer; among them, lung adenocarcinoma has also become the most common pathological type. In 2015, the World Health Organization (WHO) integrated multidisciplinary research on lung adenocarcinoma and revised its classification criteria, classifying lung adenocarcinoma into atypical adenomatous hyperplasia (AAH·carcinoma in situ), adenocarcinoma in situ (AIS), minimally adenocarcinoma, (MIA), and invasive adenocarcinoma (IAC); among them, atypical adenomatous hyperplasia and carcinoma in situ are classified as preinvasive lesions. With the continuous improvement of imaging equipment, technology and diagnostic capabilities, and the wide application of low-dose chest thin-layer CT for lung cancer screening, the detection rate of early-stage lung adenocarcinoma with ground-glass nodule (GGN) as the main manifestation has been greatly improved. Ground-glass nodules refer to nodules with a diameter of less than 30 mm and increased cloud-like density on CT thin-layer lung window images, with clear or blurred boundaries, and the original blood vessels and bronchial shadows in the nodules can still be identified. During the pathological progression of lung adenocarcinoma from preinvasive lesions to invasive lung adenocarcinoma, CT images can all appear as ground-glass density nodules, which lack specificity. According to relevant statistics, the 5-year disease-free survival rate of patients with preinvasive lesions after wedge resection is 100%. For patients with minimally invasive lung adenocarcinoma, precise resection of lung segments or subsegments has a 5-year survival rate after surgery, which is nearly 100%. However, patients with invasive lung adenocarcinoma need to be treated with relatively invasive lobectomy and lymph node dissection, and the 5-year survival rate after surgery does not exceed 9. Therefore, the infiltration of ground glass nodules has a crucial impact on the choice of surgical approach. The traditional CT morphological features of ground-glass nodules have always played a pivotal role in clinical diagnosis, including the size, mean cT value, shape, lobulation sign, burr sign, vacuole sign, air bronchus sign, vascular bundle sign, and pleural depression sign; however, the diagnostic value of cT signs mainly depends on the experience of the diagnostic imaging doctor; so, there is a lot of subjectivity. The features of early-stage lung cancer are often atypical, which makes the differential diagnosis of lung adenocarcinoma subtypes more difficult. Due to the heterogeneity of the tumor or the limitations of the needle biopsy, the traditional preoperative lung biopsy, it often cannot accurately reflect the overall invasiveness of the lesion. And needle biopsy is an invasive examination, which not only brings pain to the patient but also may cause complications such as bleeding and pneumothorax, and there are certain operational risks. Therefore, if the infiltration degree of ground-glass nodule-type lung adenocarcinoma can be accurately and noninvasively identified before surgery, it will have extremely important guiding significance for the precise selection of clinical surgical methods and the individualized formulation of treatment plans.

RETRACTED

## 2. Literature Review

Arai et al. said that lung cancer is currently the malignant tumor with the highest morbidity and mortality in the world [1]. Liu et al. said that the American Cancer Society predicts that there will be about 230,000 new cases in the United States in 2018, and the death toll from lung cancer will also be as high as 154,000, ranking first in the incidence and mortality of malignant tumors [2]. Babiy et al. said that the latest statistics in China in 2017 showed that the number of lung cancer cases was 730,000, the number of deaths was 590,000, and the two figures also topped the list [3]. Choi et al. said that known risk factors for lung cancer include smoking and air pollution, and the incidence of lung cancer is increasing year by year with the increase of tobacco abuse and environmental pollution worldwide [4]. Blackstone and El-Aini stated that surgical resection is the preferred treatment for early stage lung cancer, and it is mainly treated by a combination of surgery, radiotherapy, and chemotherapy [5]. Wang et al. said that in recent years, the statistics of lung cancer pathological types showed that lung adenocarcinoma has replaced lung squamous cell carcinoma as the type with the highest incidence and thus has received extensive attention [6]. Yuan et al. said that the three authoritative organizations of the International Association for the Study of Lung Cancer/American Thoracic Society/European Respiratory Society jointly released a new version of the pathological classification of lung adenocarcinoma in 2011, canceling the original “bronchioalveolar carcinoma (BAC)” statement, put forward new concepts such as “adenocarcinoma in situ (AIS” and “minimally invasive carcinoma (MIA”), and refined the diagnostic types of lung adenocarcinoma [7]. Shenoy et al. stated that lung adenocarcinoma has no specific symptoms in the early onset and is easily overlooked. When hemoptysis, chest pain, and other related symptoms appear, it means that the disease course has entered an advanced stage [8]. Qiu et al. said that the five-year survival rate of patients with stage IA lung adenocarcinoma can reach 90,070, and that of stage IB is 73,070. Most of the early-stage patients with pathological types have a good prognosis, but more than 20% of patients still have adverse prognostic events, such as local recurrence and distant metastasis [9]. The prognosis of patients with intermediate and advanced lung adenocarcinoma is generally poor. CT of early-stage lung adenocarcinoma can manifest as ground-glass density nodules (GGNs), which can be refined into pure ground-glass nodules (GGNs) by the presence or absence of solid components (pGGN) and mixed ground glass nodules (mGGN). The development process of lung adenocarcinoma can be regarded as a continuous process from atypical adenomatous hyperplasia (AAH) to invasive adenocarcinoma (IAC), and pGGN has a tendency to transform into mGGN. On imaging, it is generally believed that the presence of a solid component in GGN is related to the degree of infiltration, but many postoperative pathological results confirmed that pGGN appeared on CT, but the pathological results were infiltrative lesions. At present, the clinical tendency is to carry out long-term follow-up or limited lung resection for preinfiltrating lesions, in order to preserve more healthy lung tissue. Perre et al. say that preserving healthy lung tissue as much as possible can help patients recover from postoperative pulmonary function, especially in the elderly or patients with extremely poor cardiopulmonary function, and it is of great significance to improve the quality of life after surgery [10]. For invasive lesions, lobectomy and enlarged lymph node dissection should be selected more carefully to avoid the risk of postoperative recurrence and metastasis. And there is evidence that invasive adenocarcinoma has a higher risk of recurrence after surgery than noninvasive adenocarcinoma. If it is possible to determine whether there is infiltration of pGGN by CT examination, it can avoid the psychological burden and economic pressure brought by long-term follow-up observation to a certain extent and can also guide the clinical practice of timely surgical resection of invasive lesions, so as to avoid delaying the prognosis caused by the disease; in the process of diagnosis and treatment of lung cancer, CT has an irreplaceable status, no matter from the detection of the disease or the review during treatment. Currently, HRCT is more recommended for pulmonary GGN scanning, its advantage is that HRCT uses thin-layer bone algorithm scanning, which can display the fine structure of the lung more clearly, and HRCT is available in 512 × 512 or 1024 × 1024 matrix with spatial resolution in the range of 0.12-0.35 mm. It has definite advantages in showing the edge of the lesion, the internal structure, and the relationship with the small blood vessels and bronchioles. At the same time, compared with conventional chest CT examination, it is more accurate in distinguishing the nature of nodules, especially in distinguishing the degree of infiltration of nodules. However, it is difficult for doctors to evaluate CT images with the naked eye to obtain the information contained in the pixels. Under such a background, the emergence of radiomics is expected to change this situation. Radiomics collects medical image information, extracts high-throughput data from it, and conducts in-depth mining of quantitative data to obtain quantitative information. In the era of advocating precision medicine, traditional medical imaging is highly subjective and provides limited quantitative information. Radiomics quantifies image data, the extracted nodule feature information far exceeds the signs obtained by naked eye observation and has high repeatability, and some of the obtained information has the predictive ability of tumor phenotype, which is in line with the concept of precision medicine. One of the key issues in radiomic analysis is the choice of a reliable and reproducible image assessment method, which requires accurate delineation of the edges of the lesion. There is a good natural contrast between lung nodules and lung fields, which can ensure accurate segmentation of lesions, making them ideal research subjects. Combining radiomics with pGGN is a noninvasive preoperative prediction of the degree of nodule invasion by automatically acquiring quantitative features of pGGN on HRCT images. At present, preoperative judgment of pGGN infiltration degree by noninvasive methods is a hot spot in foreign research. Conventional imaging diagnostic methods and radiomic methods, respectively, determine the degree of infiltration of pGGN and the excellent degree of diagnostic methods, in order to better assist clinical selection of reasonable treatment plans. By comparing the excellence of the two diagnostic methods at the same time, the authors hope to better assist the clinical selection of a reasonable treatment plan, as shown in Figure 1.

RETRACTED

## 3. Methods

Paraffin-embedded specimens obtained after surgery in all cases were sectioned with 0.4 cm thick tissue sections, including the largest cutting plane of the tumor, and tissue sections were then stained with hematoxylin and eosin. All sections were studied by 2 pathology professors. When there is a dispute, the seniority in pulmonary pathology is taken as the standard. All cases were diagnosed and classified according to the WHO classification of lung adenocarcinoma, and the types of pathological diagnosis included the following: MIA and IAC. IHC staining was performed with Ki-67 protein antibody (Santa Cruz Biotechnology, Santa Cruz, CA, USA) at a dilution of 1 : 100. Cells with brown nuclei were considered positive. Select the three regions with the highest density of positive cells. Randomly count 100 cells in each area under high magnification and calculate the percentage of positive cells as the Ki-67 index. The Ki-67 index for the three regions was calculated and averaged. Analysis was performed using SPSS 24.0 statistical software (SPSS Inc., Chicago, IL, USA). In all variables, the mean ± standard deviation was used for normal distribution, and the median was used for nonnormal distribution. The differences in clinical and imaging characteristics of the MIA group and IAC group were compared. Count data were analyzed by chi-square test, measurement data with normal distribution were analyzed by Student's *t*-test, and nonnormal distribution was analyzed by Mann–Whitney *U* test. *P* value <0.05 was statistically significant [11]. A neural network model was established with variables with *P* value <0.05 in univariate analysis as input variables and factors, and the conjugate gradient optimization algorithm was used. Receiver operating characteristic curve *C*, ROC, was analyzed by MedCalc v19.0.2 software, and the area under the curve (AUC) was calculated and compared to evaluate the predictive value of IAC. A retrospective analysis was carried out in this study. Among 469 patients with pGGNs, 268 of them were MIA, and 201 were IAC. The mean age of the patients in the 0MIA group (54.90 ± 10.92 years) was lower than that in the IAC group (61.27 ± 9.12 years) (*P* ≤ 0.001) and in the MIA group. The proportion of smoking patients was less than that in the IAC group (*P* = 0.015). Gender and lesion location were not statistically different between the two groups (specifically shown in Table 1). In this study, a total of 436 pGGNs were stained with ki-67, of which 246 were in the MIA group and 190 in the IAC group [12]. The ki-67 070 of the MIA group (5.00, 5.00-7.63) was lower than that of the IAC group (5.00, 5.00-10.00; (*P* ≤ 0.001), as shown in Table 1.

In the morphological analysis of CT images, the lesions in the MIA group were more round-like than those in the IAC group (*P* = 0.036). The lesions in the MIA group had fewer imaging morphological signs (lobulation sign, vacuole sign, air bronchus sign, and vascular bundle sign) in the MIA group and in the IAC group (all *P* < 0.050) [13, 14]. In the quantitative analysis of CT images, the CT-LP and CT-W of the MIA group were lower than those of the IAC group; the diameter, volume, and mass of the MIA group were significantly lower than those of the IAC group (all *P* ≤ 0.001), as shown in Table 2.

Among the 469 pGGNs, the AUCs of CT-LP, CT-W, lesion diameter, volume, and mass to determine IAC were 0.67, 0.67, 0.78, 0.77, and 0.81, respectively, as shown in Table 3.

RETRACTED

Based on CT imaging features, the variables with *P* value <0.05 in univariate analysis were used as input variables and factors to establish a neural network model. The diagnostic performance analysis of neural network model to distinguish MIA and IAC showed that its AUC, accuracy, sensitivity, and specificity were 0.91, 83.55%, 82.09%, and 85.45%, respectively. CT-W, lesion diameter, volume, and mass showed the diagnostic efficacy of distinguishing MIA and IAC. The AUC value of the neural network model is significantly better than the latter prediction results (all *P* < 0.050), as shown in Figure 2.

WHO proposes a new classification system based on adherent growth pattern as a clinicopathological type, which clarifies the heterogeneity between different pathological types of lung adenocarcinoma, and the pathological manifestations, immunohistochemistry, growth rate, surgical plan, and prognosis were all the same; therefore, the authors retrospectively analyzed 469 pGGNs confirmed by pathology before surgery and established an effective neural network model by using thin-slice CT imaging features, and the diagnostic performance for differentiating MIA and IAC presented as pGGNs was greatly improved. In the study, the age of the patients in the MIA group (54.90 ± 10.92 years) was lower than that in the IAC group (61.27 ± 9.12 years) (*P* ≤ 0.001). In a study of 154 cases of subsolid pulmonary nodules < 5 mm, Ren et al. also found that the age of onset of MIA was lower than that of IAC (*P* = 0.015), which is basically similar to the results of this study [15]. This study also showed that the proportion of smokers in the MIA group was less than that in the IAC group (*P* = 0.015), but there was no statistical difference in gender and lesion location between the two groups. The shape and edges of pGGNs are determined by a combination of different cell growth rates and matrix responses, and most MIAs are oval (86.70070) [16]. In this study, the lesions in the MIA group were more round-like (72.76070) than in the IAC group (63.68070), which was similar to previous results. At the same time, other imaging morphological features (lobulation sign, vacuole sign, air bronchus sign, and vascular bundle sign) of pGGNs in this study were statistically different between the two groups, and the IAC group was more than the previous literature results, which is also roughly the same. The bronchus of the same order is always accompanied by the pulmonary artery, when the vascular bundle sign and the air bronchus sign appear in pGGNs, the lesion may have more blood and oxygen supply, and it may reflect the accelerated growth and infiltration of tumor cells. Pathologically, the vacuolar sign refers to obstructive expansion of small airways, multiple ruptured alveolar fusion cavities, and lung tissue not occupied by tumor tissue. However, unlike most of the previous literature, there was no statistical difference between the two groups in the pleural stretch sign in this study. Due to human factors and experience differences in the cognition of conventional imaging signs, therefore, there may also be some degree of instability. The size and CT value of the lesions are of great significance for the diagnosis and identification of pGGNs. It is generally believed that the larger the pGGNs, the higher the grade of malignancy. In this study, the diameter, volume, and mass of the MIA group were significantly lower than those of the IAC group (all *P* ≤ 0.001). Using quantitative CT histogram and FDG-PET analysis of 225 cases of c-0/I stage lung adenocarcinoma, it was found that the tumor diameter and volume in the IAC group were higher than those in the preinvasive lesion group. Meng's analysis of 145 cases of GGNs also showed that the tumor in the IAC group was significantly larger than that in the MIA group (12.84 vs. 9.0 scm, *P* < 0.05). It can be seen that the size of pGGNs is a more important distinguishing indicator. The CT value of the lesion can reflect more tumor cells growing along the alveolar septa, there is a strong negative correlation with the air gap retained in the tumor, and the CT attenuation value increases as the infiltrating component continues to spread and grow [17, 18]. In the study of 253 pGGNs, the CT value of preinvasive lesions was lower than that of IAC (*P* = 0.020), which was similar to our results. In this study, CT-LP and CT-W were lower in the MIA group than in the IAC group (-659.45 vs. -606.44: -677.96 vs. -634.19; all *P* ≤ 0.001).

RETRACTED

## 4. Experiments and Analysis

In recent years, the popularity of spiral CT has made the detection rate of pulmonary nodules higher and higher. Compared with conventional scanning, HRCT has clear advantages in displaying the internal and surrounding characteristics of nodules. Some studies have pointed out that the probability of malignant tumor in GGN is significantly higher than that in solid nodules, and the most common pathological type is lung adenocarcinoma. There is a real component in the ground glass density, indicating that the lesion has infiltration or fibrosis, and the progression is rapid. It is recommended to reexamine in a short period of 3-6 months. After the lesion enlarges or becomes consolidated, surgical resection should be taken for treatment [19]. However, whether the pure ground glass component lesions are inflammatory lesions or tumor lesions requires further observation and judgment. And according to the new version of lung adenocarcinoma classification in 2011, the judgment of AIS and MIA must be judged by a complete gross specimen, and there is a sampling position error in needle aspiration cytology, which causes differences in pathological results. If ground glass lesions are rashly surgically removed, the postoperative pathological results are confirmed to be benign, which may lead to controversy over overdiagnosis [20]. However, some scholars have continuously found that pGGN also has invasive components, and delaying preoperative diagnosis may lead to poor long-term prognosis. The 65 nodules in this study were all surgically resected pGGN, and there were also invasive lesions such as MIA and IAC, which also confirmed the above point of view. The authors analyzed the qualitative and quantitative characteristics of pGGNs < 30 mm in diameter on HRCT. Qualitative features included lobulation sign, burr sign, vacuole sign, vascular cluster sign, and nodule size and mean CT value in quantitative features, which were statistically significant between the two groups for preinvasive and invasive lesions (*P* < 0.05). There were no significant differences in gender, lesion location, shape, air bronchus sign, pleural traction sign, and tumor-lung interface (*P* > 0.05). Studies have shown that the lobulation sign and the spicule sign are more frequently present in invasive lesions, and our findings are consistent with those reported in the literature [21]. Lobulation and spicules are the edge features of nodular lesions. Some scholars believe that the proportion of spicule signs is higher in lung adenocarcinoma; lung adenocarcinoma lesions with few solid components are more prone to lobulation signs and spicules, which is consistent with our study. The results are consistent, and it is considered to be related to the invasion of tumor cells into the interstitial structure of the lung, resulting in uneven arrangement of tumor cells and differences in tumor cell growth rates [22]. The vascular bundle sign is an independent risk factor for judging the presence or absence of infiltrating components. The biological behavior of the tumor is also confirmed by the side, the degree of malignancy is positively correlated with its ability to proliferate, and vascular endothelial factor surges in the early stage of tumorigenesis, resulting in an increase in new blood vessels or vascular remodeling. Analysis of the blood vessels in the GGN showed that the tortuosity, thickening, and aggregation of the blood vessels in the lesions increased the blood supply in the lesions, which were more likely to appear in MIA and IAC lesions, which was consistent with our results. The study found that the degree of tortuosity of pulmonary veins in MIA was higher than that of preinvasive lesions, indicating that vascular changes can distinguish preinvasive and invasive pGGN to a certain extent. The vacuolar sign refers to the nontextured area within 1-2 mm in diameter of the pulmonary nodule, the vacuolar sign may be the lung tissue that is not filled by tumor cells in the lesion or the alveolar cavity and the remnant luminal structure of the bronchioles destroyed by tumor invasion, and it has been reported in the literature that the vacuolar sign can be used in differentiating benign and benign pulmonary nodules. The degree of malignancy is significant, and there are many female patients in this study, but the gender comparison was not statistically significant between the two groups (expansion = 0.012, *P* = 0.912). At present, the incidence of lung adenocarcinoma in women is increasing year by year, especially in nonsmoking women. The cause is unknown, but it may be related to second-hand smoke and cooking fumes. Among the 65 nodules in this study, 41 cases of bilateral upper lobe lesions, accounting for 63% of the total, also showed a pattern of bilateral upper lobe predilection, but no relationship between bilateral upper lobe predisposition and pGGN was found. Relationship. In this study, no exact correlation was found between the distribution of lesions with or without invasion [23]. We divided the nodules into two groups: round/round-like and irregular. The round/round-like group was the majority (84.6%). There was no difference between the two groups (*P* = 0.555). The nodule morphology is related to benign and malignant nodules, but these conclusions are compared between the two groups of benign and malignant nodules, and this study is compared within the malignant pGGN; so, the conclusions are different. The morphology of malignant pGGN was also compared, and the conclusions obtained also support this study. There was no statistical significance in the air bronchus in this study (*P* > 0.05). It is believed that the appearance of the air bronchus sign in the lung adenocarcinoma nodule is related to the fibrosis within the lesion pulling the bronchus, but the research subjects in this study were all pGGN solid or subsolid. In terms of sexual nodules, the degree of fibrosis in pGGN lesions is lower; so, the conclusions are different. The pleural stretch sign is greatly affected by the location of the nodule, and lesions in the subpleural area are more likely to have pleural stretch signs. In this study, no definite statistical significance was found between the two groups (*P* = 0.882) [24]. The size of the nodule directly reflects the growth rate of the nodule. In this study, the average size of the nodule in the preinfiltration group was 11.16 ± 4.29 mm, and the infiltration group was 15.10 ± 5.35 mm. Previous studies have shown that the diameter of AIS in pGGN is significantly smaller than that of MIA and IAC, 10 mm was selected as the cut-off value for judging invasive lesions, and 13.6 mm was considered as the cut-off point for judging invasive lesions; there are differences in the grouping method used in this paper because of the errors caused by species or manual measurement or the classification of MIA as preinvasive lesions. Previous studies have shown that the size of CT value is considered as a method to distinguish different pathological types. The arrangement of tumor cells in invasive lesions changes. The higher the CT value, the higher the degree of malignancy. In the study, the analysis of pGGN also included the relationship between tube voltage and CT value was explored. For images scanned in the range of 120-140 kVp, the CT value was related to the degree of infiltration, while the low voltage of 40-110 kVp was not meaningful for identification. In this study, a high voltage of 140 kVp was also used for scanning, which ensured the reliability of CT value analysis. By analyzing the data, we obtained that the mean CT values of preinvasive and invasive lesions were -5 87.29 ± 78.86 HU and −494.78 ± 85.53 HU, there was a significant difference *P* ≤ 0.001, the cut-off value was -533.50 HU, and the sensitivity was 0.704 and specificity 0.763. Considering the differences in CT value measurement methods and scanning parameters, the results were basically consistent with those reported in the literature. The high-quality images of HRCT play an important role in the diagnosis of GGN, but the information obtained by radiologists from medical images is limited. There is a lot of overlap in imaging features between preinvasive lesions and invasive lesions, and it is difficult to distinguish morphologically. Traditional CT images can only obtain simple quantitative information such as nodule size and CT value. The judgment of the degree of pGGN infiltration is mostly based on clinical experience, which is prone to missed diagnosis and misdiagnosis. At present, there is no definite quantitative information to distinguish whether there is an infiltrating component in pGGN, and it can only be judged by postoperative pathology. The emergence of radiomics provides a new idea to solve this problem [25]. Radiomic analysis of pulmonary nodules has been widely concerned, and its advantages lie in improving diagnostic specificity and sensitivity while minimizing the workload of radiologists [26, 27]. Omic analysis is to extract high-throughput information from CT images and quantify it to obtain morphological features, grayscale features, and texture features, and the extraction of these features is generally done automatically by computers. In addition, by analyzing image features and clinical data, radiomics can provide additional diagnostic information for the internal components, and lymph node metastasis and distant metastasis of lung adenocarcinoma, the observation and measurement of the morphology, nodule size, and average CT value of pGGN by conventional imaging diagnostic methods are limited to the naked eye. Detailed and three-dimensional, all images are delineated layer by layer to form a three-dimensional structure, which can more fully obtain the volume and morphological characteristics of the lesion. Secondly, the first-order histogram and high-order texture features obtained through the original DICOM image are based on the changes of different grayscale values in the image, the human eye can only distinguish 16-level grayscale changes, and it is often difficult to understand subtleties; there are many omissions, the identification of image grayscale through computer software is more detailed and accurate, and the judgment of infiltration components is more accurate. However, the infiltration degree analysis and long-term prognosis evaluation of pGGN by radiomics is still in its infancy, and it has not been widely used. In the future, we will incorporate images from more sources to validate and optimize the diagnostic performance of this omics model [28].

RETRACTED

## 5. Conclusion

The qualitative and quantitative characteristics of pGGN of lung adenocarcinoma with a diameter of less than 30 mm on HRCT were analyzed by conventional imaging diagnostic methods, and it was found that lobulation sign (*P* ≤ 0.001, burr sign (*P* = 0.008), vacuole sign (*P* = 0.047, vascular sign), cluster sign (*P* = 0.001), nodule size (*P* = 0.001), and mean CT value (*P* ≤ 0.001) were meaningful in distinguishing preinvasive and invasive lesions. The optimal cut-off values of nodule size and mean CT value were, respectively, 12.7 mm and -544.50 HU. The DICOM images of lung adenocarcinoma pGGN with HRCT diameter < 30 mm were analyzed by the radiomic method, the quantitative features of medical image data were deeply excavated to obtain two omics parameters of “dimension” and “sphericity,” which were used to establish a group, a scientific model was established, and the validation of the model was meaningful for diagnosing the degree of pGGN infiltration. The quantitative diagnostic value of radiomics (AUC = 0.824) was higher than that of conventional imaging diagnostic methods (AUC = 0.740 and 0.784).

## Figures and Tables

**Figure 1:** The diagnostic effect of CT radiomic features in pulmonary invasive mucinous adenocarcinoma.

**Figure 2:** ROC curve analysis for predicting pGGN as IAC.

**Table 1:** Summary of basic clinical data of the MIA group and IAC group.

Variable	All (*n* = 469 example)	MIA (*n* = 268 example)	IAC (*n* = 201 example)	*P*
Age				0.00
Mean ± standard deviation	57.63 ± 10.67	54.90 ± 10.92	61.27 ± 9.12	
Gender				0.90
Male (example)	146 (31.13%)	75 (27.99%)	71 (35.32%)	

**Table 2:** Differences of CT imaging features between the MIA group and IAC group.

Variable	All (*n* = 469 example)	MIA (*n* = 268 example)	IAC (*n* = 201 example)	*P*
Lesion shape				0.036
Round shape (example)	323 (68.87%)	195 (72.76%)	128 (63.68%)	
Irregular shape (example)	146 (31.13%)	73 (27.24%)	73 (36.32%)	
Lobography (example)	165 (35.18%)	81 (30.22%)	84 (41.79%)	0.010
Vacuolation sign (example)	84 (17.91%)	39 (14.55%)	45 (22.39%)	0.029
Air bronchus sign (example)	87 (18.55%)	41 (15.30%)	46 (22.89%)	0.037
Vascular bundle sign (example)	178 (37.95%)	53 (19.78%)	118 (58.71%)	≤0.001

**Table 3:** Diagnostic efficacy of quantitative imaging parameters of lesions in the MIA group and IAC group.

	AUC	95% CI	Optimal value	Sensitivity	Specificity
CT-LP, HU	0.67	0.62~0.71	-633.93	66.20%	61.90%
CT-W, HU	0.67	0.62~0.72	-656.28	61.70%	66.00%
Diameter, mm	0.78	0.74~0.82.	1.35	77.60%	65.70%
Volume, mm^3^	0.77	0.73~0.81	681.30	78.10%	63.40%
Mass, mg	0.81	0.78~0.85	213.76	85.10%	63.80%

## Data Availability

The data used to support the findings of this study are available from the corresponding author upon request.

## References

[1] Arai K., Iwasaki T., Tsuchiya C., Sonoda A. (2020). Annexin a2 expression in the aerogenous spread of pulmonary invasive mucinous adenocarcinoma with gastric lineage. *Case Reports in Oncological Medicine*.

[2] Liu J., Zhang S., Luo J. (2020). Prognosis of early stage pulmonary mucinous adenocarcinoma with different treatments. *Translational Cancer Research*.

[3] Babiy Y., Sychova T., Dykan I. (2019). Radiological aspects of the new "international multidisciplinary classification of lung adenocarcinoma": methodological bases and own experience. *Radiation Diagnostics Radiation Therapy*.

[4] Choi Y., Kim K. H., Jeong B. H. (2020). Clinicoradiopathological features and prognosis according to genomic alterations in patients with resected lung adenocarcinoma. *Journal of Thoracic Disease*.

RETRACTED

[5] Blackstone N., El-Aini T. (2021). Medical image of the month: mucinous adenocarcinoma of the lung mimicking pneumonia. *Southwest Journal of Pulmonary and Critical Care*.

[6] Wang L., Hirano Y., Heng G., Ishii T., Yamaguchi S. (2020). Mucinous adenocarcinoma as a high-risk factor in stage ii colorectal cancer: a propensity score-matched study from Japan. *Anticancer Research*.

[7] Yuan H. J., You Z. B., Li G. Y. (2020). Clinical characteristics and treatment strategies of prostatic mucinous adenocarcinoma: a report of 10 cases and literature review. *National Journal of Andrology*.

[8] Shenoy V., Buckley M., Hosseini H., Ma M., Aggarwal A. (2020). S1710 signet ring cell mucinous adenocarcinoma of the colon manifesting as intermittent hiccups. *The American Journal of Gastroenterology*.

[9] Qiu T., Ru X., Yin K., Yu J., Song Y., Wu J. (2020). Two nomograms based on ct features to predict tumor invasiveness of pulmonary adenocarcinoma and growth in pure ggn: a retrospective analysis. *Japanese Journal of Radiology*.

[10] Perre S. V., Duron L., Milon A. (2021). Radiomic analysis of htr-dce mr sequences improves diagnostic performance compared to bi-rads analysis of breast mr lesions. *European Radiology*.

[11] Li M., Chen T., Zhao W., Wei C., Shen J. (2020). Radiomics prediction model for the improved diagnosis of clinically significant prostate cancer on biparametric mri. *Quantitative Imaging in Medicine and Surgery*.

[12] Liu Z., Jiang Z., Meng L., Yang J., Zhou R. (2021). Handcrafted and deep learning-based radiomic models can distinguish gbm from brain metastasis. *Journal of Oncology*.

[13] Chen J. M., Wan Q., Zhu H. Y., Ge Y. Q., Ding Z. M. (2020). The value of conventional magnetic resonance imaging based radiomic model in predicting the texture of pituitary macroadenoma. *Zhonghua Yi Xue Za Zhi*.

[14] Montrucchio G., Lupia T., Lombardo D. (2021). Risk factors for invasive aspergillosis in icu patients with covid-19: current insights and new key elements. *Annals of Intensive Care*.

[15] Ren X., Li C., Ma X. (2021). Design of multi-information fusion based intelligent electrical fire detection system for green buildings. *Sustainability*.

[16] Shriram S., Jaya J., Shankar S., Ajay P. (2021). Deep learning-based real-time AI virtual mouse system using computer vision to avoid COVID-19 spread. *Journal of Healthcare Engineering*.

[17] Roy K., Jana S., Ghosh S. K., Mahanty B., Mandal D. (2020). Three-dimensional MOF-assisted self-polarized ferroelectret: an effective autopowered remote healthcare monitoring approach. *Langmuir*.

[18] Xin L., Jianqi L., Jiayao C., Fangchuan Z., Chengyu M. (2021). Study on treatment of printing and dyeing waste gas in the atmosphere with Ce-Mn/GF catalyst. *Arabian Journal of Sciences*.

RETRACTED

[19] Avc A., Korkut M., Bekta A. F., Syüncü S. (2020). Thoracic fluid content measurement: diagnostic value of suspected pulmonary oedema in acute decompensate heart failure. *Eurasian Journal of Emergency Medicine*.

[20] Huang R., Zhang S., Zhang W., Yang X. (2021). Progress of zinc oxide-based nanocomposites in the textile industry. *IET Collaborative Intelligent Manufacturing*.

[21] Pegoraro J. A., Lavault S., Wattiez N., Similowski T., Gonzalez-Bermejo J., Birmelé E. (2021). Machine-learning based feature selection for a non-invasive breathing change detection. *Bio Data Mining*.

[22] Chu Z. G., Li W. J., Fu B. J., Lv F. J. (2020). Ct characteristics for predicting invasiveness in pulmonary pure ground-glass nodules. *American Journal of Roentgenology*.

[23] Gu J., Wang W., Yin R., Truong C. V., Ganthia B. P. (2021). Complex circuit simulation and nonlinear characteristics analysis of GaN power switching device. *Nonlinear Engineering*.

[24] Ylmaz F. H., Tarak N., Gültekin N. D., Yücel M., Altunhan H. (2021). Comparison of the efficacy of three natural surfactants in preterm turkish newborns with respiratory distress syndrome. *The Journal of Pediatric Research*.

[25] Brunlich J., Kppe-Bauernfeind N., Petroff D., Franke A., Wirtz H. (2022). Nasal high-flow compared to non-invasive ventilation in treatment of acute acidotic hypercapnic exacerbation of chronic obstructive pulmonary disease—protocol for a randomized controlled noninferiority trial (elvis). *Trials*.

[26] Khader M. M., Bishawi A. A., Kambal A., Abdelmajid A. (2020). Sars-cov-2 infection presenting as colitis with chest and abdomen ct findings. *Radiology Case Reports*.

[27] Jansson-Knodell C. L., Harris C. E., Loftus E. V., Walker R. C., Virk A. (2021). Histoplasmosis in inflammatory bowel disease with tumor necrosis factor-alpha inhibitors: safe to continue biologics?. *Digestive Diseases and Sciences*.

[28] Cheng W., Li Z., Zhu Y., Ding N., Yi H. (2021). Surgical correction for scimitar syndrome by right thoracotomy and direct anastomosis in children. *Pediatric Investigation*.

